The article "High-Quality Nursing Care for the Elderly in the Department of Otolaryngology" was retracted in 2023. Reasons: signs of a paper mill; suspected computer-generated content; unreliable results or conclusions; concerns about the data.

# High-Quality Nursing Care for the Elderly in the Department of Otolaryngology

**DOI:** 10.1155/2021/5542562

**Published:** 2021-04-19

**Authors:** Yeping Huang, Huili Chen

**Affiliations:** ^1^Department of Otorhinolaryngology, People's Hospital of Zhuji City, Zhuji, Zhejiang 311800, China; ^2^Zhongnan Hospital of Wu Han University, Wuhan, Hubei 430071, China

## Abstract

ENT patients have different types of diseases and clinical symptoms, and generally, patients have a low level of understanding of their professional knowledge about their ENT diseases. In this paper, quality nursing interventions in otorhinolaryngology require nursing staff to implement relevant nursing interventions in the process of implementing relevant nursing care, which should be based on patients' needs, and guide patients to perform rehabilitation exercises according to their individual conditions, in addition to establishing continuous nursing interventions with patients at the time of discharge with the help of modern technology. By comparing the nursing satisfaction of patients in the observation group and the control group, it was found that the nursing satisfaction of patients in the observation group who received humanistic nursing was higher, and the difference was statistically significant compared with that of the control group (*P* < 0.05). The SCL-90 scale scores of patients in both groups were not significantly different on the day of admission as verified by *t* values, and the SCL-90 scale scores of patients in both groups changed to a certain extent after hospitalization. The difference between the two groups was verified by *t* value.

## 1. Introduction

With socioeconomic development and increased demand for medical care, the need to provide better and better nursing care has become a new nursing requirement. Evidence-based nursing refers to the careful, accurate, and wise application of the best currently available research basis by nursing staff, followed by the development of a valuable, credible and complete care plan based on the nursing staff's own acquired knowledge, skills, and clinical work experience, taking into account the patient's values, wishes, and actual situation. Evidence-based nursing, developed on the basis of traditional nursing concepts, is a branch of evidence-based medicine, and evidence-based nursing is considered to be the best nursing approach at this stage and has gained importance in various departments [1–5]. Patient safety has emerged as one of the great challenges facing healthcare in the 21st century [6]. Given its importance to the health system and its impact on society as a whole, it has now become a focus of discussion both nationally and internationally [7]. General surgery is the mother of all subdisciplines in the modern surgical field and, as the largest specialty in the surgical system, it has a wide spectrum of diseases and covers many organs, involving liver, biliary tract, pancreas, gastrointestinal, anorectal, and vascular diseases, tumors of the thyroid and breast, and traumatic injuries, and is mainly treated surgically. In recent years, the rate of population aging has accelerated and the number of elderly surgical patients has increased rapidly [8].

The article "High-Quality Nursing Care for the Elderly in the Department of Otolaryngology" was retracted in 2023. Reasons: signs of a paper mill; suspected computer-generated content; unreliable results or conclusions; concerns about the data.

Surgical patients are prone to various unsafe events after surgery due to a series of blows such as anesthesia and surgery. Among them, there is a category of “potentially critically ill” patients, whose condition is not very serious on the surface, and there is no obvious clinical manifestation of a specific organ failure, but if the condition of these patients is neglected and effective interventions are not taken in time, it is likely that their condition will deteriorate rapidly within a few hours or days and turn into critically ill patients and even endanger their lives [9]. Ensuring patient safety is the first element of hospital safety management, and it is also a prerequisite and the most basic requirement for improving the quality of medical services. For nursing, providing an effective and reasonable level of supervision is the focus of medical safety work. However, due to the limited medical resources, how to effectively manage critically ill patients or potentially critically ill patients outside the intensive care unit area has become an urgent concern for healthcare professionals [10]. In addition, how clinical healthcare professionals can quickly and accurately determine the criticality of a patient's condition and the magnitude of potential risk still largely relies on individual healthcare professionals' knowledge and clinical experience and lacks quantitative and standardized objective indicators, resulting in patients receiving inappropriate monitoring during hospitalization, which can lead to misdiagnosis, missed diagnosis, and even delayed conditions, resulting in adverse events, medical disputes, and waste of medical resources. The introduction of the early warning scoring system has enabled the ward nurses to be more proactive in identifying the condition, and the nurses can select the appropriate interventions according to the “trigger value” and summon the doctors or relevant specialists through the “call doctor criteria,” which greatly improves the safety of patients. Therefore, it is imperative to predict early changes in the condition of postsurgical patients and to establish a scientific, effective, and standardized early warning monitoring program for timely intervention [11]. Most patients show obvious signs such as shortness of breath, altered state of consciousness, arrhythmias, abnormal blood pressure, low arterial oxygen saturation, and abnormal urine output several hours before admission to the intensive care unit or the occurrence of cardiac arrest [12]. A large observational study of hospitalized patients showed that 9% of patients had at least one abnormal vital sign at the beginning of their admission. More than 80% of patients were fully identifiable within the first 24 hours of deterioration but failed to receive timely and effective interventions because nurses failed to monitor vital signs in their entirety and report these conditions to physicians in a timely manner. Many patients are admitted to the ICU because they fail to receive monitoring and treatment consistent with the acute and critical nature of their condition, resulting in their exacerbation [13].

The article "High-Quality Nursing Care for the Elderly in the Department of Otolaryngology" was retracted in 2023. Reasons: signs of a paper mill; suspected computer-generated content; unreliable results or conclusions; concerns about the data.

Evidence-based nursing initially originated from evidence-based medicine, and then with the development of evidence-based medicine and the inspiration of ideas, the nursing discipline also began to adopt the approach of evidence-based medicine and the concept of evidence-based nursing emerged. Traditional nursing is disease-centered nursing, while evidence-based nursing is person-centered, so nursing thinking is completely different from traditional nursing. The urgent nursing problem of the ENT patient is the lack of knowledge of the patient's disease, the risk of airway obstruction, pain, negative psychological emotion, and lack of patient compliance, and the relevant literature search was carried out on the above problem, and 22 literature papers were selected to be highly scientific and reliable to create and personalize nursing plans, combining them with patient needs. The study showed that the observation group improved the rate of patients' health knowledge and satisfaction rate of nursing care. The SAS, SDS, and VAS scores of patients in the observation group were lower than those in the control group after care, and patient compliance was better than that in the control group, showing that evidence-based care is effective and more suitable for clinical care. In conclusion, the use of evidence-based nursing in ENT nursing can better solve the nursing problems that patients need to solve, and the nursing effect is better than traditional nursing methods.

### 1.1. Related Works

Patients with nasopharyngeal carcinoma often have two or more stable symptoms that coincide, interact, and influence each other as a cluster of symptoms that affect the patient's quality of life. In the sleep disorder symptom cluster, cancer and its treatment modalities can affect sleep quality, which can lead to depressed mood and reduced cognitive function [14]. In contrast, studies have shown that sleep disorders have negative effects on physical, cognitive, and motor function in individuals diagnosed with cancer. These negative responses may lead to interruptions in treatment, thereby prolonging overall treatment, which has been shown to have a detrimental effect on overall survival. In the oral dysfunction group, oral mucositis, oropharyngeal soreness, swallowing/chewing difficulties, taste abnormalities, and salivary thickening have a common mechanism of action, leading to reduced eating, resulting in decreased body mass, a pronounced sense of morbidity, reduced willingness to socialize, and severe negative emotions such as anxiety and depression [15].

The article "High-Quality Nursing Care for the Elderly in the Department of Otolaryngology" was retracted in 2023. Reasons: signs of a paper mill; suspected computer-generated content; unreliable results or conclusions; concerns about the data.

In some nasopharyngeal cancer survivors, dental shutdown and dry mouth are chronic problems that may lead to malnutrition. Depression in cancer patients was also found to be significantly and positively correlated with their malnutrition, and patients' depression may reduce their desire to eat, thereby affecting their nutritional status. Poor nutritional status during treatment is a significant predictor of mortality in HNC, and its adverse consequences also include impaired immune function, reduced vitality, and decreased resistance to the disease, which leads to increased morbidity and increased complications due to the side effects of treatment [16]. In order to better manage patients to improve their nutritional status, reduce psychological burden, decrease the incidence of complications, and improve their survival and quality of life, it is necessary for clinical staff to develop a holistic patient-specific care plan based on careful assessment of patients to improve their physical and psychological functioning and ensure adequate nutritional intake [17]. Not only should the overall condition of patients with nasopharyngeal carcinoma be carefully assessed prior to the start of radiation therapy, a care plan should be developed and followed up to prevent complications related to functional impairment and malnutrition in patients with NPC undergoing radiotherapy, but longitudinal changes occurring during and after treatment should also be closely followed and aimed at developing relevant interventions to prevent and reduce long-term radiotherapy-related complications and malnutrition. Therefore, there is an urgent need to establish a well-established and effective continuum of care program to provide guidance and follow-up throughout the different time points of diagnosis, treatment, and recovery, which will help to reduce the occurrence of complications and improve survival and quality of life [18].

The article "High-Quality Nursing Care for the Elderly in the Department of Otolaryngology" was retracted in 2023. Reasons: signs of a paper mill; suspected computer-generated content; unreliable results or conclusions; concerns about the data.

The use of conventional continuity of care is highly discretionary, with an incomplete care program, lack of relevance, and no timely and effective evaluation and feedback mechanisms. Case management is widely used in the healthcare service industry as a cost-effective strategy for coordinating individual health needs, bridging the gaps in routine continuing care. It includes the management of a wide range of chronic diseases, such as hypertension, chronic obstructive pulmonary disease, and breast cancer, and has been used with significant success in practice. Researchers conducted a randomized controlled trial with 12-month follow-up in a primary care clinic in southern Brazil, where adult hypertensive patients were randomly assigned to an intervention group (*n* = 47) and a usual care group (*n* = 47), with case management consisting of care consultations, telephone contact, home visits, health education, and appropriate referrals, with care plans modified as necessary, resulting in case management. The intervention group with case management was more effective in controlling hypertension than the control group and improved in waist circumference, weight, and treatment compliance compared to the control group [19].

A study of 103 patients with chronic obstructive pulmonary disease (COPD) found that patients who went through a case management intervention had a significantly higher quality of life than the control group [20]. Researchers randomized 335 women aged 65 years and older with newly diagnosed breast cancer to the control and intervention groups, including home visits, telephone conversations, meeting with cases at physician appointments, visiting cases during hospitalization, and contacting and interacting with cases at other locations in the community throughout the intervention period, and found that, compared to the control group, women in the case-managed intervention group were significantly more likely than controls to have normal or near-normal range of motion in the arm on the side of their breast cancer for 2 months after surgery. The researchers randomly assigned 95 patients who had just completed cancer treatment to 11 cancer centers in the canton of Zurich, Switzerland. Patients in the case management group met with a case manager at least three times over a 12-month period and were assessed on the basis of patient-reported outcomes and it was found that case management improved quality of life, reduced the burden of returning to normal life for cancer patients, and met the needs of early cancer survivors for ongoing care. Researchers interviewed healthcare professionals after implementing oncology case management in a tertiary oncology specialty medical institution and found that oncology case management helped to improve the doctor-patient relationship and enhance healthcare professionals' operational competencies [21]. In a randomized controlled trial in Denmark, 280 colorectal cancer patients were assigned in a 1 : 1 ratio to either the control group or the case management (CM) intervention group. 30 weeks after patient recruitment, an interim pilot questionnaire was sent to all patients' GPs and the responses of GPs in both groups were compared, resulting in GPs' appreciation of case management. Patients in the intervention group had significantly less contact with the hospital. Case management of nasopharyngeal carcinoma has been reported in China to improve patients' level of hope and self-efficacy, increase the rate of first follow-up and implementation of established treatment plans, and benefit patients, but the model of case management of nasopharyngeal carcinoma differs from one to another, with a single follow-up approach, a short duration, and a lack of systematic construction and validation and similarity to extended care services.

The article "High-Quality Nursing Care for the Elderly in the Department of Otolaryngology" was retracted in 2023. Reasons: signs of a paper mill; suspected computer-generated content; unreliable results or conclusions; concerns about the data.

## 2. Application of Precision Information Management in Clinical Care

### 2.1. Early Warning Score

There is a group of patients who are easily overlooked in clinical practice. They are apparently not seriously ill and do not have obvious clinical manifestations of a specific organ failure, but if they do not receive timely and effective interventions, they are likely to experience rapid changes in their condition within a short period of time and become critically ill or even their life becomes threatened. For this reason, healthcare professionals in various countries have been exploring various early warning scoring systems to quickly and accurately assess patients' conditions and identify potential risks at an early stage. Among them, the calibrated MEWS is gaining attention and recognition among healthcare professionals because of its easy availability, simple and quick assessment method, and high sensitivity in predicting changes in patients' conditions, as shown in Figure 1. Some researchers have compared the MEWS with the calibrated MEWS and found that the calibrated MEWS is more recommended for clinical use.

At the end of the 20th century, due to a severe lack of medical resources in the UK, critically ill patients were unable to receive proper placement and timely and effective intensive care, resulting in a series of medical errors. In order to improve the situation, the UK government asked clinical staff to establish a faster and more convenient scoring system to help them identify the disease risk of critical patients early, so as to provide reasonable early medical intervention for patients with a certain risk index as soon as possible. To this end, the UK government has established the Patient at Risk Emergency Team to comprehensively assess the condition of “potentially critically ill” patients and recovering patients and to provide timely medical intervention or referral to a more appropriate medical unit. The early warning score (EWS) was first proposed by researchers and then, after extensive clinical research, the early warning score based on the EWS was endorsed by the National Health Service (NHS) in the United Kingdom as a method of assessing patients' conditions in healthcare settings. It was subsequently recommended and used by the British Intensive Care Society and the Royal College of Physicians of London to assess the risk of patients on integrated wards. A Severity of Illness Scoring Group, established by the NHS in the UK, developed the SEWS, which researchers applied to 848 acutely admitted patients and found that the SEWS was better able to identify high-risk patients. EWS and MEWS were gradually introduced into China and are widely used in emergency medicine, ICU wards, internal medicine, and other areas. Researchers added oxygen saturation to MEWS to form the corrected MEWS and compared MEWS with the corrected MEWS and found that the corrected MEWS was more accurate and sensitive than MEWS in assessing the condition and prognosis of patients with “potentially critical illness” in prehospital emergency. The accuracy and sensitivity of the calibrated MEWS were found to be better than the MEWS in assessing the condition and prognosis of “potentially critically ill” patients in prehospital emergency.

The article "High-Quality Nursing Care for the Elderly in the Department of Otolaryngology" was retracted in 2023. Reasons: signs of a paper mill; suspected computer-generated content; unreliable results or conclusions; concerns about the data.

The MEWS is an objective index tool for early identification of patients' risk of deterioration, and the patient's condition is evaluated by scoring 5 indicators and assigning a certain score to physiological indicators within a certain range (Table 1), among which the AVPU scoring method is used for scoring the state of consciousness. The correction of the MEWS score is based on the content of the MEWS score, with the addition of the important physiological parameter index of blood oxygen saturation, whose reference range is ≥95%; 91% to 94% for mild hypoxemia; 85% to 90% for moderate hypoxemia; and <85% for severe hypoxemia.

### 2.2. Scoring Methodology for Quality Care

In the corrected MEWS, temperature parameters were assigned a score in the range of 0 to 2. Respiratory rate, systolic blood pressure, heart rate, consciousness, and oxygen saturation were assigned a score in the range of 0 to 3. The total score was obtained by adding up the scores of individual parameters according to the parameter table, with the lowest score being 0 and the highest score being 17. The higher the total score, the more severe the condition. The scoring is done mainly by nurses. The scoring interval is related to the optimal trigger value for correcting the MEWS score. Some investigators used the following scoring interval: after the patient is admitted to the hospital, the nurse starts scoring and dynamically monitors the patient's vital signs every 4 h for a score of 1 to 3; every hour for a score of 3 on any single variable; every 30 min for a score of 3 to 5; and every 15 min for a score of 6 and above. Vital signs are monitored every 15 min for a score of 6 and above. The scoring system is easy to use, and medical staff can quickly obtain the relevant index parameters at the bedside and complete the patient scoring and condition assessment within minutes, as shown in Figure 2.

Nurses can take appropriate action with patients based on optimal trigger values and a specially tailored early warning process. Applying the corrected MEWS to 300 prehospital emergency patients, researchers found that a corrected MEWS score of 5 or more increased the likelihood of patient admission to the ICU, and a corrected MEWS score of 8 or more increased the risk of patient death. Using the corrected MEWS, researchers retrospectively analyzed 171 patients admitted to a specialty inpatient unit after surgery on a surgical ward and found that the corrected MEWS was highly accurate in predicting patient transfer to the ICU, with a cutoff point of 5 being optimal: with a corrected MEWS score of 5 or less, most patients were treated in the surgical inpatient unit; with a score of 5 or more, patients were potentially at risk for change. Patients with a score of 5 or higher are potentially at high risk for change and need to be admitted to the ICU for treatment and increased level of care. The researchers applied the corrected MEWS to 275 patients with acute poisoning and found that a corrected MEWS score of ≥5.5 was the optimal cutoff point for criticality in patients with acute poisoning. Currently, most of the studies on the corrected MEWS score have been used clinically for acute and critical care, prehospital emergency care, pretest triage, and postoperative patient transport. Some scholars have explored the combined application of the corrected MEWS score with the addition of some relevant important physiological parameters, and some scholars have also explored the comparison between the corrected MEWS score and the MEWS score.

The article "High-Quality Nursing Care for the Elderly in the Department of Otolaryngology" was retracted in 2023. Reasons: signs of a paper mill; suspected computer-generated content; unreliable results or conclusions; concerns about the data.

### 2.3. Experimental Design

Sixty-four patients, 31 males and 33 females, aged 21–69 years with a mean age of 45.3 years, who were hospitalized for ear, nose, and throat diseases between September 2015 and September 2020 were selected. The primary diseases were mainly nasal polyps, chronic rhinitis, tonsillitis, rhinorrhea, otitis media, and acute laryngitis. The patients were randomly divided into observation group and control group, 32 cases each. In the observation group, there were 16 males and 16 females, aged 44.8 ± 12.0 years; in the control group, there were 15 males and 17 females, aged 45.5 ± 11.0 years, as shown in Table 2. The differences between the two groups in terms of gender, age, and disease type were not statistically significant (*P* < 0.05) and were comparable.

Patients in the control group were given conventional nursing care, including keeping the ward environment quiet, advising patients to get more rest, eating a diet with easily digestible food, and controlling the occurrence of infection complications. The observation group implemented evidence-based care on the basis of the control group, which mainly consisted of finding urgent nursing problems, and the nursing staff of the department searched for urgent nursing problems according to the type of disease and nursing experience and the needs of patients and categorized them as follows.

#### 2.3.1. Care of Patients with Inadequate Knowledge of the Disease

After the patient is admitted to the hospital, we explain the relevant disease knowledge for the disease suffered and the treatment to prevent recurrence. For example, patients with chronic rhinitis should wear masks when going out in cold weather, avoid going to crowded areas as much as possible, etc. The causes of persistent rhinorrhea are more complicated, and once bleeding occurs, first apply local pressure to stop bleeding on your own and call medical personnel quickly, etc.

#### 2.3.2. Care for the Risk of Airway Obstruction

Reasonable treatment measures should be taken immediately for acute laryngitis, and nursing staff should strengthen inspection, 1 time/30 min, and pay more attention to patients prone to tracheal tube dislodgement and take strengthening fixed intubation.

#### 2.3.3. Pain Care

For pain care, the ward can be configured with newspapers, play soft music, read newspapers, and listen to music to divert attention; do not let the patient endure in case of heavy pain; timely report to the doctor to be given appropriate analgesic drug intramuscular injection to reduce the patient's pain.

#### 2.3.4. Care of Negative Psychological Emotions

Patients were psychologically assessed upon admission, and psychological assessment was performed with the Self-Assessment Scale for Anxiety (SAS) and the Self-Rating Scale for Depression (SDS) to find out patients' psychological problems. Nursing staff should work in an amiable and enthusiastic manner, learn to think differently about patients with more obvious psychological problems, and actively give psychological support.

The article "High-Quality Nursing Care for the Elderly in the Department of Otolaryngology" was retracted in 2023. Reasons: signs of a paper mill; suspected computer-generated content; unreliable results or conclusions; concerns about the data.

#### 2.3.5. Care of Patients with Inadequate Compliance

We should explain to patients the possible consequences of inadequate compliance and encourage them to cooperate with medical staff in all medical and nursing treatments and also explain to their families and friends so that they can obtain more social support and improve compliance.

We observed the improvement of SAS and SDS scores, patients' knowledge of disease health, patients' satisfaction with nursing care, treatment and nursing care compliance, and pain level using visual analog score (VAS) before and after nursing care in both groups.

1. SAS scale: there are 20 items with 4 levels under each item, and a score of <50 is normal, with higher scores indicating more severe anxiety.
2. SDS scale: there are 20 items, and a score of <53 is considered normal, with higher scores indicating more pronounced depressive symptoms.
3. Pain level: the VAS visual analog scale was used, with 11 levels from 0 to 10, with higher scores representing more severe pain.
4. Patients' compliance with treatment and care: we designed our own assessment criteria, including whether patients could take medication on time, whether they could cooperate with treatment, and whether they could cooperate with care. Adherence was scored on a scale of 1 for not at all, 2 for occasionally, 3 for basically, and 4 for completely.

The statistical analysis was performed using SPSS 17.0 statistical software, and the measured data were expressed as (*x* ± *s*) using *t* test, and the count data were expressed as (%) using *χ*2 test, and the difference was considered statistically significant at *P* < 0.05.

## 3. Results and Analysis

### 3.1. Comparison of Nursing Information Management and Satisfaction

The knowledge rate of ENT diseases in the observation group was 84.38% higher than that of the control group, 46.88% (*χ*2 = 9.97, *P*=0.008), and the satisfaction rate of patient care in the observation group was 93.75% higher than that of the control group, 68.75% (*χ*2 = 6.56, *P*=0.018); see Figure 3.

Evidence-based nursing originally originated from evidence-based medicine, and later, with the development of evidence-based medicine and the inspiration of ideas, the nursing discipline also began to adopt the approach of evidence-based medicine, and the concept of evidence-based nursing emerged. Traditional nursing is disease-centered care, while evidence-based nursing is people-centered, so nursing thinking is completely different from traditional nursing. Evidence-based nursing consists of three main elements: the basis of nursing research, the personal skills and level of nursing staff, and the actual situation and wishes of the patient. (2) A literature search is conducted to find valuable and credible literature on the problem. (3) The value of the retrieved information is evaluated by nursing staff with expertise in the field. (4) Develop a plan that incorporates the screened and valuable empirical literature and the patient's needs. (5) Begin implementation of the care plan and assess the effectiveness of implementation through dynamic observation.

The article "High-Quality Nursing Care for the Elderly in the Department of Otolaryngology" was retracted in 2023. Reasons: signs of a paper mill; suspected computer-generated content; unreliable results or conclusions; concerns about the data.

The urgent care problems of ENT patients are the lack of patients' knowledge about their diseases, the danger of airway obstruction, pain, negative psychological emotions, and the lack of patient compliance, so we conducted a literature search for the above problems, selected 22 literature papers with high scientific credibility, and combined them with patients' needs to develop an individualized care plan. The study showed that the observation group improved the rate of patients' health knowledge and satisfaction rate of nursing care. The SAS, SDS, and VAS scores of patients in the observation group were lower than those in the control group after care, and patient compliance was better than that of the control group, showing that evidence-based care is effective and more suitable for clinical care, as shown in Figure 4.

The calibrated MEWS is an objective tool for early identification of patients at risk of deterioration. In this study, we used the calibration MEWS used at Freeman Hospital in the United Kingdom and combined it with information technology and embedded it in an electronic nursing documentation system to achieve a simple and rapid application for early warning monitoring of the condition of patients undergoing general anesthesia and to objectively assess the degree of criticality and the potential risk of deterioration of the patient's condition by scoring the patient's pulse, systolic blood pressure, respiratory rate, body temperature (axillary temperature), consciousness, oxygen saturation (with sufficient oxygen), and urine output. Seven indicators are scored to enable early and objective quantitative assessment of the criticality of patients after general anesthesia and the presence of potential risks. Studies have demonstrated the ability of the calibrated MEWS score to determine the criticality of patients and to identify “potentially critically ill” patients. The corrected MEWS score is a tool used by health professionals to identify clinical deterioration of a patient's condition and can be considered a safety barrier in care, in addition to complementing clinical judgment. This study found that the early warning monitoring program, which clarifies the trigger criteria and interventions for nursing staff at all levels of monitoring precautions, can guide nurses to take appropriate interventions in a timely manner according to the scoring results and has been recognized by nursing managers and clinical nurses. In this study, it was found through interviews with nurses that nurses can assess patients' vital signs directly at the bedside with the help of the corrected MEWS score and that, after combining it with informatization, it can be imported directly into the paperwork records automatically, avoiding duplication of work and improving work efficiency to a certain extent, as shown in Figure 5. Therefore, the informatization-based condition alert monitoring program based on calibration of MEWS can be applied to postoperative patients in general surgery.

The article "High-Quality Nursing Care for the Elderly in the Department of Otolaryngology" was retracted in 2023. Reasons: signs of a paper mill; suspected computer-generated content; unreliable results or conclusions; concerns about the data.

This study analyzed the occurrence of nursing adverse events in both groups, mainly including misaspiration, catheter slippage or blockage, unscheduled extubation, and fluid extravasation. The results of the study showed that the information-based condition alert monitoring program based on the corrected MEWS reduced the incidence of nursing adverse events (*P* < 0.005) and, at the same time, improved physician satisfaction with nursing care (*P* < 0.005) and patient satisfaction with nursing care (*P* < 0.005). This is consistent with the findings of Schwartz et al. [20]. As the condition of elderly patients after surgery is highly variable and the morbidity and mortality rate are high, early detection of changes in patients' condition and implementation of dynamic monitoring and effective intervention can effectively reduce or eliminate the occurrence of nursing adverse events and maximize patient safety. In contrast, it is often difficult for nurses to make a comprehensive and dynamic assessment of patient condition changes through clinical work experience.

Based on the calibration of MEWS, the information-based condition alert monitoring program sets different frequencies of vital signs monitoring for patients with different levels of monitoring, enabling nurses to dynamically understand changes in patients' conditions, grasp the criticality of patients' conditions, and motivate nurses to take the initiative to observe conditions and care. The information-based condition early warning monitoring program can accurately identify changes in patients' conditions and can also automatically pop-up boxes to remind nurses to take appropriate interventions to adopt the appropriate level of monitoring and timely management of patients' conditions, thus reducing the occurrence of nursing adverse events and improving patient satisfaction. With the help of corrected MEWS scores, it provides nurses with an objective basis for condition assessment, enabling nurses to provide objective data support when communicating with doctors about their conditions, promoting effective communication between doctors and nurses about changes in patients' conditions, and greatly increasing doctors' satisfaction with the work of nursing staff, as shown in Figure 6. The nurses also provided suggestions for the improvement of the information system: sound reminders and eye-catching signs should be added to the early warning reminder function to strengthen the reminders, and the connection with the doctor's side can promote the joint discovery of changes in the patient's condition by the doctors and nurses.

The article "High-Quality Nursing Care for the Elderly in the Department of Otolaryngology" was retracted in 2023. Reasons: signs of a paper mill; suspected computer-generated content; unreliable results or conclusions; concerns about the data.

### 3.2. Analysis of Experimental Results

Patient condition monitoring is one of the important duties of nursing staff. At present, the clinical workload is large and junior nurses undertake a large amount of nursing work, but their relatively low mastery of professional knowledge and insufficient work experience lead to weak foresight of condition changes as well as observation ability, problem identification, and problem solving. The corrected MEWS score, as an objectified condition early warning scoring system, overcomes the defects of previous nursing staff's reliance on subjective judgment for condition observation, enables rapid and accurate identification of patients' conditions, and helps nursing staff obtain real-time and dynamic information about patients' condition changes. In this study, with the advantages of accuracy, efficiency, and convenience of computers, the corrected MEWS score was embedded into the nursing information system, and the corresponding parameters were automatically matched and the score was calculated, which not only can give full play to the advantages of high condition recognition of the corrected MEWS score and achieve dynamic assessment of the condition changes of elderly postoperative patients, but also avoid the risk of incorrect judgment of the condition due to manual calculation errors and improve the accuracy of the assessment. It improves the accuracy of assessment, reduces the nursing workload, and also provides strong support for nurses to dynamically monitor the changes in patients' conditions. The results of this study found that the informatization-corrected MEWS scoring system was able to reduce the postoperative vital sign monitoring of patients, but the difference was not statistically significant (*P* < 0.05), as shown in Figure 7. Qualitative interviews with nurses also revealed that the application of the informational condition warning monitoring program based on the corrected MEWS can help nursing staff to dynamically monitor changes in patients' conditions without increasing the nursing workload.

The article "High-Quality Nursing Care for the Elderly in the Department of Otolaryngology" was retracted in 2023. Reasons: signs of a paper mill; suspected computer-generated content; unreliable results or conclusions; concerns about the data.

Corrected MEWS scores provide a rapid and accurate quantitative assessment of the criticality of a patient's condition and help nursing staff obtain real-time information about changes in the patient's condition, especially potential risk events, which can prevent medical risks caused by untimely and incorrect observation and treatment, thereby shortening the patient's hospital stay and improving the operational efficiency of medical resources. At the same time, due to its simplicity, easy access to information, low operating cost of its system, and not being limited by the hardware and equipment conditions of the hospital, the application of the corrected MEWS score does not require additional costs, and the informationized condition warning monitoring program based on the corrected MEWS also provides a graded monitoring program for the condition monitoring of patients after general anesthesia, ensuring that patients receive proper monitoring and treatment and avoiding unplanned transfers to the ICU. This will ensure that patients are properly monitored and treated, avoid unplanned transfers to ICU, further save medical resources, reduce patients' medical costs, and improve the rational allocation and effective utilization of medical resources. In this study, the number of cases transferred to ICU in the experimental group was less than that in the control group, but the difference was not statistically significant (*P* > 0.05), as shown in Figure 8, which was not consistent with the results of previous studies, which may be related to the exclusion of patients directly transferred to ICU after surgery when selecting the study subjects.

The application of the informatization system can improve the quality and efficiency of nurses' nursing documentation writing, effectively standardize nurses' behavior, reduce nurses' labor intensity, and improve the level of nursing documentation writing. The results of this study showed that the information-based early warning monitoring program based on the correction of MEWS can effectively improve the standardization rate of nursing records written by nurses (*P* < 0.05) and nurses' own satisfaction with nursing work (*P* < 0.05). Nursing records and condition observation are the focus of nurses' work, and improving the quality of nursing record writing is important for improving the quality of care and the level of patient safety. Writing nursing records correctly and without errors usually takes a lot of nurses' time, and errors in writing nursing records may even cause medical disputes. At present, with the clinical workload, the relative shortage of nurses, and the increase of new nurses, the level of nursing documentation writing ability varies, and the nursing documentation records lack objectivity, continuity, and completeness. The informationized early warning and monitoring program based on corrected MEWS scores provides clear pathway and standardized management of nurses' condition observation and assessment, recording frequency, and content and relies on the computer to automatically calculate corrected MEWS scores, timely reminding nurses to assess patients' conditions, ensuring complete and continuous nursing assessment and recording, effectively reducing the incidence of nursing document recording defects, and standardizing nursing. This has effectively reduced the incidence of defects in nursing documentation and standardized nursing documentation.

The article "High-Quality Nursing Care for the Elderly in the Department of Otolaryngology" was retracted in 2023. Reasons: signs of a paper mill; suspected computer-generated content; unreliable results or conclusions; concerns about the data.

## 4. Conclusion

In this paper, the nursing model used in the clinic is no longer just disease-centered, and the holistic nursing model guided by the concept of the new biological, psychological, and social medical model is applied in clinical care. In order to meet the increasing nursing needs of patients, nurses should carefully complete patient-centered holistic nursing care, paying attention to meeting both the physical and psychological nursing needs of patients and giving full play to the role of psychological nursing to keep patients in the best physical and mental state so that their resistance to disease can be improved. In this study, patients in the control group only received conventional nursing interventions, while patients in the observation group received humanistic nursing. The degree of nursing satisfaction of patients with the observation group was significantly higher than that of the control group. In conclusion, the implementation of humanistic nursing can meet the nursing needs of endocrine patients, and while giving full play to the nursing-assisted treatment, it can also better improve patients' compliance and satisfaction with nursing care, which is worth applying and promoting in the nursing care of endocrine patients.

## Figures and Tables

**Figure 1:** Early warning scoring mechanism.

**Figure 2:** Relationship between patient scores and condition assessment and time.

**Figure 3:** Comparison of patients' health knowledge and nursing satisfaction between the two groups.

The article "High-Quality Nursing Care for the Elderly in the Department of Otolaryngology" was retracted in 2023. Reasons: signs of a paper mill; suspected computer-generated content; unreliable results or conclusions; concerns about the data.

**Figure 4:** Comparison of SDS, SAS, VAS, and compliance scores between two groups of patients.

**Figure 5:** Efficiency comparison under MEWS scoring mechanism.

**Figure 6:** Caregiver satisfaction improvement.

**Figure 7:** Automatic matching of care information systems.

**Figure 8:** Comparison of patients' subsequent disease progression.

**Table 1:** Correction of modified early warning scores.

No.	Index	−2	−1	0	1	2
1	Pulse (times/min)	<40	41–60	61–70	71–80	>80
2	Systolic pressure (mmHg)	<70	71–90	91–110	111–190	>190
3	Respiratory rate (times/min)	<10	11–20	21–30	31–40	>40
4	Body temperature (°C)	/	<35	36–40	41–45	>45
5	AVPU	/	/	Awake	Voice	Painful

**Table 2:** Selecting patient information.

Group	Average age (years old)	Gender (male/female)	Course of disease (month)	Injury part	
				Left	Right
Control	44.8 ± 12. 0	16/16	2–13	18	22
Observation	45.5 ± 11.0	15/17	2–13	18	22

## Data Availability

Data sharing is not applicable to this article as no datasets were generated or analyzed during the current study.
